# Review on the Application of Metalearning in Artificial Intelligence

**DOI:** 10.1155/2021/1560972

**Published:** 2021-07-05

**Authors:** Pengfei Ma, Zunqian Zhang, Jiahao Wang, Wei Zhang, Jiajia Liu, Qiyuan Lu, Ziqi Wang

**Affiliations:** ^1^College of Science, North China University of Science and Technology, Tangshan 063210, China; ^2^School of Metallurgy and Energy, North China University of Science and Technology, Tangshan 063210, China

## Abstract

In recent years, artificial intelligence supported by big data has gradually become more dependent on deep reinforcement learning. However, the application of deep reinforcement learning in artificial intelligence is limited by prior knowledge and model selection, which further affects the efficiency and accuracy of prediction, and also fails to realize the learning ability of autonomous learning and prediction. Metalearning came into being because of this. Through learning the information metaknowledge, the ability to autonomously judge and select the appropriate model can be formed, and the parameters can be adjusted independently to achieve further optimization. It is a novel method to solve big data problems in the current neural network model, and it adapts to the development trend of artificial intelligence. This article first briefly introduces the research process and basic theory of metalearning and discusses the differences between metalearning and machine learning and the research direction of metalearning in big data. Then, four typical applications of metalearning in the field of artificial intelligence are summarized: few-shot learning, robot learning, unsupervised learning, and intelligent medicine. Then, the challenges and solutions of metalearning are analyzed. Finally, a systematic summary of the full text is made, and the future development prospect of this field is assessed.

## 1. Introduction

In the context of the development of big data, the emergence of machine learning algorithms has a milestone significance in data mining. In the past, artificial intelligence lacking the support of big data, as a kind of machine intelligence designed to imitate human cognitive functions [1], could not achieve the effect of intelligence due to the slow processor speed and small amount of data, but today big data provides massive amounts of data for artificial intelligence [2], so that artificial intelligence technology can achieve real intelligence. The close integration of big data and artificial intelligence is an important milestone in the progress of human history, and it also makes the public more and more concerned with artificial intelligence technology [3]. However, with the advent of the era of artificial intelligence, the development of machine learning has encountered many challenges, including issues such as increased demand for decision-making, prediction efficiency, and prediction accuracy. In addition, successful cases are mainly concentrated in the areas where a large amount of data can be collected or simulated and areas where a large amount of computing resources can be used, excluding many areas where data is scarce or expensive or where computing resources are unavailable [4].

In order to break through these limitations, both commercial machine learning users and big data mining tool users urgently need an algorithm that can learn models and predict independently, so metalearning (ML) came into being. Chan and Stolfo [5] used four inductive learning algorithms: ID3 (iterative dichotomizer 3) [6], CART (classification and regression trees) [7], WPEBLS (weighted parallel exemplar-based learning system) [8], and Bayes [9] to experiment on the DNA splice junction dataset (splice junction, SJ) [10], using combination strategies, arbitration strategies, and mixed strategies. The results showed that metalearning methods could improve the prediction accuracy of SJ data and was more effective than non-metalearning methods. At the same time, traditional artificial intelligence methods use fixed learning algorithms to solve tasks from scratch. On the contrary, metalearning aims to improve the learning algorithm itself based on the experience of multiple learning situations [11]. This “learning to learn” [12] approach provides opportunities to solve many traditional challenges of machine learning, including data and computing bottlenecks, as well as generalization [4].

As a kind of neural network model, metalearning provides a reliable and innovative method for solving the problems faced by machine learning in big data, and its current development momentum has been very rapid. This article aims to conduct inductive analysis and provide new insights for the application of metalearning in the field of artificial intelligence. This research reviews, analyzes, and classifies existing metalearning research to provide detailed insights into the most advanced metalearning algorithms and determine future research directions, so as to provide a comprehensive reference for the application of metalearning algorithms in the future, especially in the field of artificial intelligence.  Section 2 of this article first introduces the research process and basic theory of metalearning, and then it discusses the comparison between metalearning and traditional machine learning and the research direction of metalearning in big data.  Section 3 summarizes the application examples of metalearning in the field of artificial intelligence: few-shot learning, robotic learning, unsupervised learning, and intelligent medicine.  Section 4 discusses the challenges and solutions that metalearning faces in the field of artificial intelligence, from the two aspects of technology and application.  Section 5 encapsulates the content of the full text to make a systematic summary and outlook.

## 2. Basic Theoretical Knowledge of Metalearning

### 2.1. The Research Process of Metalearning

With the advancement of artificial intelligence technology, metalearning has experienced three stages of development. The beginning of the first development stage of metalearning can be traced back to the early 1980s, when Maudsley put forward the concept of “metalearning” for the first time and regarded metalearning as the synthesis of hypothesis, structure, change, process, and development. He describes it as “the process by which learners become aware of and begin to control their already internalized perception, research, learning, and growth habits.” In 1985, Biggs [13] used metalearning to describe the specialized application of metacognition in student learning and believed that metalearning is a subprocess of metacognition. In 1988, Adey and Shayer [14] combined metalearning with physics and proposed a new method of physics teaching based on metalearning ideas.

In the early 1990s, the development of metalearning entered the second stage, the concept of metalearning began to slowly penetrate into the field of machine learning, and many researchers contributed to the early work of metalearning in the second stage of development. As for the issue of algorithm selection at that time, some researchers have discovered that this issue is actually a learning task, and because of this, it has gradually developed in the machine learning discipline, and a brand-new field, “metalearning field,” has gradually formed [15]. In 1990, Rendell and Cho [16] innovatively proposed a method to characterize classification problems with metalearning as the idea and conducted experiments to verify that these features have a positive impact on algorithm behavior. However, this idea was mostly used in psychology at that time. In 1992, Aha [17] further expanded the metalearning idea: for a given dataset with characteristics *C*_1_, *C*_2_,…, *C*_*n*_, the rule of rejection algorithm A2 and selection algorithm A1 is obtained by selecting the rule-based learning algorithm, and this idea was first applied to the field of machine learning. In 1993, Chan and Stolfo [18] proposed that metalearning is a general technology that can combine multiple learning algorithms and used metalearning strategies to combine classifiers calculated by different algorithms. Experiments show that metalearning strategies and algorithms are more effective than other experimental strategies and algorithms. In 1994, with the European development of a large-scale classification algorithm comparison project—STATLOG (comparative testing of statistical and logical learning) [19]—as a by-product of the project, the metalearning idea has gradually attracted the attention of many scholars. In 1998, VanLehn [20] discussed how to extend metalearning to the solution of tutoring problems.

In the 21st century, more and more researchers in the field of machine learning have paid more attention to the application of metalearning ideas for algorithm selection, and the development of metalearning has also entered the third stage. In 2000, Bensusan et al. [21] used the typed high-level inductive learning framework they developed to propose metalearning based on inductive decision trees. In 2002, Vilalta and Drissi [22] proposed that metalearning and basic learning are different in the scope of adaptation levels; metalearning studies how to dynamically select the correct bias by accumulating metaknowledge, while the basis of basic learning is a priori fixed or user parameterized. At the Knowledge Discovery Conference (KDC) in 2001, an important research question, “depending on data to automatically select data mining parameters and algorithms,” fully embodies the idea of metalearning; this topic was brought up again by Fogelman at the Knowledge Discovery Conference in 2006. In 2017, Finn et al. [23] innovatively proposed a model-agnostic metalearning (MAML) algorithm, which is compatible with any model trained with gradient descent and is suitable for a variety of different learning problems, including classification, regression, and reinforcement learning. In 2019, Xu et al. [24] proposed a model-agnostic metalearning method based on weighted gradient update (WGU-MAML), which can be combined with any gradient-based reinforcement learning algorithm to improve sample efficiency. The core idea of this method is that, after updating the model parameters within a size of a few gradient steps, a set of sufficiently sensitive model parameters that can effectively adapt to multiple new tasks is found. The experimental results show that this method significantly improves the performance of the pure deep reinforcement learning algorithm, and it is superior to other existing metalearning algorithms when solving new tasks. In 2020, Xu et al. [25] proposed a few-shot network intrusion detection method based on metalearning framework and verified through experiments that the method is versatile and not limited to specific attack types, with an average detection rate of 99.62%. At the same time, Raghu et al. [26] proposed an almost no inner loop (ANIL) algorithm on the basis of model-agnostic metalearning in 2020. This algorithm has better computational performance than model-independent metalearning whether in standard image classification or reinforcement learning benchmarks, and it is found through experiments that feature reuse is the dominant factor in the effectiveness of model-agnostic metalearning. The research process of metalearning is shown in Figure 1.

### 2.2. Basic Theory of Metalearning

Metalearning is difficult to define, and even in contemporary neural network literature, metalearning is used in a variety of inconsistent ways [4]. However, metalearning can be broadly defined as learning from the information generated by the learner, which is regarded as the learning of metaknowledge of the learned information. Common deep learning models are designed to learn a mathematical model for prediction, and metalearning is not for the results of learning, but the process of learning. It is not learning a mathematical model directly used for prediction, but learning “how to learn a mathematical model faster and better.”

The algorithm flow is shown in Figure 2. The purpose here is to explore the diversity of multiple learning algorithms through metalearning, so as to improve the accuracy of prediction. This is achieved through a basic configuration with several different basic learners and a metalearner who learns from the output of the basic learner. Metalearners can use the same algorithm or completely different algorithms in the basic learners, and each basic learner is provided with a complete training set of original data. However, the training set of the metalearner is generated and merged by different algorithm model tasks, which is different from the original training set. Each basic learner generates a basic classifier, and a metalearner generates a metaclassifier. Furthermore, the metalearner is not designed to pick the “best” basic classifier; on the contrary, it tries to include each classifier, that is, the prediction accuracy of the entire system is not limited to the most accurate basic classifier. The ultimate goal is to generate an overall system that performs better than the underlying base classifier.

### 2.3. Comparison of Machine Learning and Metalearning

The purposes of machine learning and metalearning are different. Machine learning aims mainly to find a classification function *f* based on data; this classification function is actually an algorithm or network designed by CNN (convolutional neural networks) etc. After training, the output parameter *θ* is used to determine such an *f*, which is

(1) $$\begin{array}{c} f\left(\text{task}\right)=\theta . \end{array}$$

Metalearning is looking for an *F*, which is a learning algorithm. Through this *F*, it is trained on a bunch of tasks to generate the parameters *θ* that we need. When encountering a new classification task, let *θ* be adjusted to the best *θ*^*∗*^ suitable for the new task and classification model and corresponding to *f*^*∗*^, namely,

(2) $$\begin{array}{c} F\left(\text{tasks}\right)=\theta ,\\ \theta \left(\text{a new tasks}\right)⟶\theta^{*}. \end{array}$$

In Figure 3, it can be clearly seen that the purposes of machine learning and metalearning are different. Machine learning is more inclined to learn directly from data and get the final prediction result, but metalearning hopes to master the abilities of learning independently and predicting new tasks according to a part of dataset.

The training process of machine learning and metalearning is also very different. The training process of machine learning is also relatively simple, just preparing the required training materials and test materials, as shown in Figure 4. However, in the metalearning training process, what needs to be prepared is not training data and test data, but training tasks and test tasks. Each task contains training data and test data, as shown in Figure 5.

Whether it is the purpose of learning or the training process of data, machine learning appears to be relatively singular, while metalearning is more extensive. Metalearning builds a large-scale framework to enable machine learning algorithms to train and predict autonomously in this framework. Therefore, metalearning can also adapt to some complex learning processes faster and is a more advanced and intelligent method, which is in line with the development trend of artificial intelligence.

### 2.4. The Research Direction of Metalearning in Big Data

With the continuous popularity of metalearning algorithm, people's research on it is also expanding in all directions, so its research direction has gradually become more complex and diverse. According to the findings of this article, the research directions of existing metalearning algorithms in big data can be roughly divided into the following three categories.

#### 2.4.1. Classifier-Based Metalearning

Classification is a very important method of data mining [27]. The concept of classification is to learn a classification function or construct a classification model on the basis of existing data, which is commonly referred to as a classifier. This function or model can map the data records in the database to a given category, so that it can be applied to data prediction. In short, the classifier is a general term for the methods of classifying samples in data mining, including algorithms such as decision trees, logistic regression, naive Bayes, and neural networks [28]. Classifier-based metalearning is just a process of learning from the basic classifier, and the input of metalearning here is also the output of the ensemble member classifier [29]. The goal of metalearning ensemble is to train an original classifier that combines the predictions of the ensemble members into a single prediction. At the same time, ensemble members and metaclassifiers need to be trained to create similar sets. The main principle of the TUPSO integration scheme is to use metalearning technology to combine multiple and possibly different single-class classifiers [29]. The metaclassifier is equivalent to a class classifier and learns a classification model containing metafeatures from metainstances. However, for those integration schemes that are particularly dependent on certain performance indicators, such as weighted performance and scoring, it is difficult for many integration schemes, including metaclassifiers, to achieve better performance.

#### 2.4.2. Metric-Based Metalearning

Metric-based metalearning refers to learning a metric space to make the learning in the space extremely efficient. This method is mostly used for small sample learning. The key is to learn an embedded network so that the original input can be converted into a suitable representation and to compare the similarity between the sample instance and the instance under test. Sung et al. [30] proposed to model a relation network that contains both embedding modules and relation modules. The embedding module is responsible for feature extraction of the image to be tested and the sample image, while the relation module is responsible for comparing the similarity of the extracted features to directly determine which category the image to be tested belongs to. This method directly uses neural network learning metrics, and in this process, the training is carried out in the way of metalearning. In addition, Koch et al. [31] proposed a prototypical network to learn a metric space, in which each class has metadata, and achieved the most advanced results on the CUB-200 (Caltech-UCSD Birds 200) dataset. At the same time, Vinyals et al. [32] proposed the metric learning method of Siamese neural network. Snell et al. [33] put forward a new matching network with the idea of metric learning based on deep neural features, which can train mechanism through its corresponding metric. Garcia and Bruna [34] defined a novel metric method for graph neural network architecture. These metric-based algorithms can also be used to implement the metalearning training process, because this type of algorithm can more appropriately represent data features to learn better, and thus can achieve better learning performance. However, for tasks such as regression and reinforcement learning, these algorithms have not been proven to achieve the same effect, so further in-depth research is needed.

#### 2.4.3. Optimizer-Based Metalearning

The optimizer-based metalearning method is to learn an optimizer; that is, one network (metalearner) learns how to update another network (learner) so that the learner can learn the task efficiently. The advantage of this method is that it allows the metalearner to independently design an optimizer to complete new tasks, eliminating the need for manual debugging of some optimizers such as Adam [35]. That is, the metalearner can autonomously choose a suitable optimizer by learning the experience of previous tasks, so that the model can learn new tasks efficiently and quickly. Andrychowicz et al. [36] used long short-term memory (LSTM) to replace the traditional optimizer in order to optimize a suitable optimizer for new tasks in a gradient descent manner. Since the Hessian matrix of the loss function is in an ill-conditioned state, the performance of the one-step algorithm will be greatly reduced. Therefore, Park and Oliva [37] proposed to learn a local curvature information matrix in the metalearning process to realize the transformation of the gradient in space, so that the transformed gradient has better generalization performance for the new task. The traditional optimizer only guarantees that the loss of the current step is smaller than the loss of the previous step, and only focuses on the benefit of the current cycle, which is seriously lacking in integrity. The metalearning optimizer can coordinate the impact of multiple steps in the future on the current step, achieve the effect of looking forward and looking backward, and find the current strategy that has the best impact on future results. However, when faced with large networks or complex optimization problems, the optimization cost of the metalearning optimizer is very demanding, and its performance stability may be relatively poor.

As shown in Table 1, this section mainly analyzes and compares the main research directions of metalearning in big data from the three directions of classifier, metric, and optimizer. Metalearning of each research direction requires us to grasp its advantages and strive to explore reasonable solutions to its shortcomings, so as to give full play to its respective advantages in the future application of artificial intelligence. In general, regardless of the direction of metalearning in big data, it is hoped that it can achieve the purpose of autonomous training and problem-solving, which not only improves training efficiency, but also reduces the process of human participation, which is a major advancement in artificial intelligence. However, the current research on these directions still lacks further practice, so that it cannot be fully applied in many fields and solve some complex and diverse problems. Therefore, this study suggests that it is necessary to conduct more in-depth exploration in these directions in the future.

## 3. Specific Analysis of the Application of Metalearning in the Field of Artificial Intelligence

Since entering the new era of big data, artificial intelligence has been widely used in people's lives; no matter it is work, study, or entertainment, it cannot be separated from artificial intelligence [38]. The production and application of artificial intelligence technology have not only enriched people's lives, but also improved work efficiency, leading to significant development of more new machine learning technologies [39].

With the idea of metalearning being put forward, it has been widely applied. As mentioned in the research process in Section 1, the application of metalearning involves fields such as pedagogy, psychology, and physics, but most of the applications in these fields are still stuck in the exploratory stage. With metalearning and machine learning beginning to merge with each other after a large number of applications in the field of artificial intelligence, driven by big data, the public's understanding of metalearning began to gradually expand from theories, models, and algorithm steps to applications. This section mainly focuses on four aspects: few-shot learning, robot learning, unsupervised learning, and intelligent medicine, to conduct a detailed overview and analysis of the application of metalearning in the field of artificial intelligence based on big data.

### 3.1. The Field of Few-Shot Learning

With the hot development of large-scale neural networks, the drawbacks of their performance being limited by the size of the training set have gradually emerged. If the training set contains too few samples, network overfitting will occur, making it difficult to realize the potential of deep networks. Therefore, the application of metalearning in few-shot learning is gradually being valued by people, and it is widely used in this field. Recently, there are many few-shot learning methods that can match metalearning in terms of image classification task performance, but they are only designed for classification and are not easy to use for object detection tasks. For example, Wang et al. [40] combined metalearning and face recognition and proposed a new face recognition method based on metalearning, called meta-face recognition (MFR) method. This method uses the combination of gradient and metagradient to update the model, so as to achieve the effect of improving the model generalization performance; the experimental results show the versatility and optimality of the method.

Metalearning technology uses metaknowledge accumulated from historical tasks as prior knowledge, then learns a small number of target samples to quickly master new tasks, effectively improves training methods and training time, and has strong adaptability and robustness to unknown scenarios. Therefore, the few-shot learning technology based on metalearning is also widely used in scenes such as classification [41, 42], target detection [43, 44], and video synthesis [40]. In these scenarios, new categories of samples are often scarce or difficult to obtain. In addition, various factors in practical applications are also much more complicated than experiments. Some actual data to be tested are also volatile, which may lead to the situation where the data differs from the training data. For traditional machine learning algorithms, especially deep learning-based methods, a large-scale labeled training set is required when learning a new task, even if the model is pretrained on other classification problems, so it is more difficult to apply in the above scenarios. However, contrary to traditional machine learning algorithms, metalearning aims to deal with the problem of data limitation when learning new tasks. Therefore, in the application process of the above-mentioned few-shot learning, the dependence on the number of target samples will also be greatly improved. It avoids the problems of parameter overfitting and low model generalization performance, has greater adaptability to unknown conditions, and provides a reliable solution for areas where samples are scarce.

### 3.2. The Field of Robot Learning

In the field of robotic learning, which is currently developing rapidly [45], the application prospects of metalearning are also very broad. Especially in terms of robot operation skills, metalearning, as a “learning to learn” method, has made good progress [46]. With the development of robot technology in the fields of home, factory, national defense, and outer space exploration [47], the autonomous operation ability of robots has attracted more attention from the public, and it is expected that it can replace humans in more complex multidomain operation tasks. However, the current methods for robots to learn operating skills are still relatively backward methods, requiring a lot of time, manpower, and cost, and are in a relatively weak stage of intelligence. Improving the ability of robots to learn operating skills autonomously and quickly is a major issue in the field of robot learning problem [48]. Finn et al. [49] proposed a meta-imitation learning (MIL) method by extending model-agnostic metalearning to imitation learning. This method allows robots to master new skills with only one demonstration, which improves robot learning efficiency, whether in simulation or in visual demonstration experiments on a real robot platform; the ability of this method to learn new tasks has been verified, and it is far superior to the latest imitation learning methods. Yu et al. [50] proposed a domain-adaptive metalearning (DAML) method based on metalearning, allowing the learning of cross-domain correspondences, so that robot learners can visually recognize and manipulate new objects after only observing a video demonstration of a human user and achieve the effect of one-time learning. Metalearning can not only help robots to imitate learning, but also cultivate the ability of robots to learn to learn. Nagabandi et al. [51] proposed a meta-reinforcement learning method that enables the robot to quickly adapt to unknown conditions or sudden and drastic changes in the environment online, and verified the effective adaptability of the model through experiments; it is especially important in the real world.

### 3.3. The Field of Unsupervised Learning

In recent years, due to the nature of unsupervised learning that can train models without supervision, it has attracted the attention of many scholars, but unsupervised learning has the characteristics of training samples without labels, so that many machine learning algorithms that are practical in unsupervised learning application becomes very difficult. However, in the field of unsupervised learning, the application of metalearning has achieved very good results, especially in training unsupervised learning algorithms. Garg and Kalai [52] proposed a meta-unsupervised-learning (MUL) framework and simplified unsupervised learning to supervised learning by considering the distribution of unsupervised problems, thereby greatly improving the performance of unsupervised learning and helping to solve different representations and questions from different fields. Based on metalearning, Li et al. [53] proposed a novel metalearning noise-tolerant (MLNT) training method, which enables the model to learn from noise-labeled data without supervision, and proved that this method has more superior performance compared with the latest technical methods through experiments.

### 3.4. The Field of Intelligent Medicine

With the gradual shortage of pathologists worldwide and the scarcity of data in the medical field, progress in the medical field is particularly important [54]. Although many scholars have tried to apply traditional machine learning algorithms to the medical field [55], in actual operation, they will always encounter many problems, such as the inability to fully integrate the algorithm into it or the inability to obtain accurate prediction results. Metalearning, however, can fill these gaps, so it has become increasingly popular in fields such as medical image classification and drug discovery. In [56], Altae-Tran et al. combined LSTM with graph neural networks to predict the behavior of molecules, such as its toxicity, in a one-time data mechanism. In [57], MAML can be adapted to weakly supervised breast cancer detection tasks, and the order of the tasks is selected according to the course, rather than randomly selected. MAML is also combined with a denoising autoencoder for medical vision question answering [58], and learning to weigh support samples as done in [59] can be applied to pixel weighting to handle skin lesion segmentation tasks with noisy labels [60].

At the same time, Nguyen et al. [58] proposed a novel visual question answering (VQA) framework for medical care, which overcomes the limitations of labeled data. Moreover, by combining the advantages of an unsupervised denoising autoencoder (DAE), which can take advantage of a large number of untagged images, with the advantages of supervised metalearning, which can learn metaweights with limited tagged data to quickly adapt to VQA problems, a small sample set can be used to train the proposed framework. The experiment proved that this method is better than the current medical visual solution method.

As shown in Table 2, the application of metalearning in artificial intelligence based on big data can well solve the bottleneck encountered in the development of artificial intelligence, which will also be a huge turning point for artificial intelligence. In addition to the above-mentioned fields, this study found that metalearning can also be applied in domain generalization [61], quantitative network, automatic speech recognition [62], and other fields, and it has great potential to be developed in many fields supported by big data.

## 4. Challenges and Countermeasures of Metalearning

Metalearning has a long history and has become more and more important in recent years. As many people have advocated, it is the key to the realization of artificial intelligence in the future [63]. In particular, the ability of metalearning to learn in each task it proposes and at the same time accumulate knowledge about the similarities and differences between tasks, is considered to be essential for improving artificial intelligence. Although the metalearning method is efficient and widely applicable, it also has many limitations. Especially in terms of technology and application, it is still facing severe tests. This section mainly summarizes the bottlenecks encountered by metalearning in terms of technology and application and, based on our research, gives corresponding countermeasures.

### 4.1. Technical Aspects

First of all, this method generally requires more similar tasks for metatraining, so the cost is higher. At present, each training task is generally modeled by low-complexity basic learners (such as shallow neural networks) to prevent the model from overfitting, so it is impossible to use deeper and more powerful architectures. For example, for the dataset miniImageNet, model-agnostic metalearning uses a shallow CNN with only 4 CONV layers, but its best performance is obtained after learning 240,000 tasks [64]. At the same time, Brock et al. [65] proposed a method for training proxy models, and Lee et al. [66] proposed to accelerate metatraining through a closed solver in the inner loop, but the effect is also very insignificant. Secondly, although the existing model can show fast and efficient learning ability on simple new tasks such as moving and sorting targets, the learning ability shown on some complex new tasks such as action cohesion is very unsatisfactory. Finally, the current algorithms are basically learning single metaknowledge, and metaknowledge is diverse, so the generalization of the model may be affected to a certain extent.

### 4.2. Application Aspects

On the one hand, although the metalearning algorithm only needs a small amount of new sample data, the data demand for similar historical tasks is very large, and the acquisition process is even more difficult. This may result in the use of a small number of fixed adjustment steps to train the weights in the learning process, so that overfitting may occur at this stage, and many gradient steps will actually increase the test error of a new task. On the other hand, the current models basically perform experiments under the condition that the distribution of new tasks and historical tasks is the same. However, due to the variability of the actual input process and the unknowability of practical applications, the new tasks and historical tasks are different from each other, and there will inevitably be errors in the distribution. This situation will not only lead to a significant reduction in the model's ability to learn new tasks, but also affect the performance of the model during cross-task learning.

### 4.3. Responses

Many scholars in the field of metalearning are very concerned about the above two challenges and believe that these two challenges may become the key to the universal application of metalearning in the field of artificial intelligence. Through our research, we found that these challenges can be solved using the following countermeasures.

In terms of technology, first of all, researchers can start with the training model of the specific task and improve the training performance of the model through gradient optimization, algorithm step improvement, and other methods, so that the model can better avoid training losses and reduce the need for metatraining tasks, thereby increasing the speed of metatraining. Secondly, researchers should deeply study the process of task execution and explore various laws in the process, especially the continuity law of action execution, so as to improve the ability of action cohesion in the process of complex task execution and improve the learning ability of the model for complex new tasks. Finally, researchers should try to combine complex and diverse metaknowledge, divide them into certain categories according to specific situations, and systematically study these metaknowledge uniformly, so as to make them better in model performance and improve the generalization performance of the model.

For applications, on the one hand, researchers can consider starting from the scale of the data and build a platform that can collect training tasks in various fields. When encountering similar available tasks, researchers can directly obtain them from this platform, avoiding the waste of time and financial resources caused by the process of obtaining data. This can not only provide sufficient historical task data for reference for the operation of the model, but also avoid the impact of overfitting and test errors on the training results. On the other hand, researchers can also refer to other machine learning and algorithms empirical methods to avoid the inconsistency of the distribution of new tasks and historical tasks and to find the integration point with metalearning, so as to solve the problem of inconsistent distribution, such as the depth-domain adaptive (DDA) method proposed by Sun and Saenko [67] and Rozantsev et al. [68] and the hybrid heterogeneous transfer learning (HHTL) algorithm proposed by Zhou et al. [69] based on deep learning.

As shown in Table 3, the current development of metalearning is mainly constrained by two levels of technology and application. In the first section of this article, the three stages of the metalearning research process have been elaborated, and the transition of each stage is the latter one. After a breakthrough in the previous stage, this breakthrough is mainly attributed to the innovative solution to the development bottleneck problem in the previous stage. After summarizing the current challenges faced by metalearning, this research believes that a new stage of metalearning research is about to come, and to achieve a leap to the new stage, it is inevitable to implement the countermeasures proposed in this research to the reality of metalearning in practical application of artificial intelligence. It is also hoped that more scholars will pay attention to these challenges in the future and propose better countermeasures to promote the development of metalearning in the field of artificial intelligence.

## 5. Summary and Outlook

In summary, in the context of big data, metalearning not only solves the problems of data, calculation, and generalization encountered by traditional artificial intelligence but also solves the problems of machine learning's prediction accuracy and efficiency in big data. Therefore, the role of metalearning in the field of artificial intelligence is more prominent. If you want to promote the all-round development of artificial intelligence in the future, you must have a clear understanding of the advantages and applications of metalearning, and it should effectively play the actual role of big data and artificial intelligence. In recent years, traditional algorithm selection and hyperparameter optimization of classic machine learning techniques (such as support vector machines, logistic regression, and random forest) have left room for metalearning. Researchers can use the same metalearning model across tasks instead of training new models for different tasks from scratch [70]. At the same time, since the birth of artificial intelligence in the 1950s, people have always wanted to build machines that learn and think about big data like humans [63]. The metalearning algorithm based on the idea that “it is better to teach him how to fish than to give him fish,” dedicated to helping artificial intelligence learn how to learn big data, is the ideal solution to realize this goal, and it is also a new generation force in the development of artificial intelligence. In the future, researchers will also make breakthroughs in a more challenging direction.

Based on the above research, it is found that the research of metalearning in the field of artificial intelligence has two aspects worthy of attention:

On the one hand, this study noticed that the current research of metalearning in the field of artificial intelligence mainly considers benchmark datasets, such as Omniglot and MiniImageNet, and fast learning, and feature reuse of metalearning on other few-shot learning datasets (such as the dataset of Triantafillou et al. [71]) will be an interesting direction in the future.

On the other hand, this study also found that, despite different views and research routes, one question remains the same: How can we use knowledge about learning (i.e., metaknowledge) to improve the performance of learning algorithms? Obviously, the answer to this question is the key to progress in this field and will continue to be the subject of in-depth research.

To sum up, this article takes the artificial intelligence based on big data as the background, introduces the research process and basic concepts of metalearning, expounds the difference between metalearning and traditional machine learning and its current main research directions in big data, and then summarizes four typical application examples of metalearning in the field of artificial intelligence: few-shot learning, robotic learning, unsupervised learning, and intelligent medicine. The future challenges and countermeasures of metalearning are analyzed and discussed from the two aspects of technology and application. This article believes that, in future research, the field of artificial intelligence and metalearning methods will be more closely integrated, which will also make daily life more intelligent in the future.

## Figures and Tables

**Figure 1:** The development of metalearning.

**Figure 2:** Flowchart of metalearning algorithm.

**Figure 3:** Machine learning vs metalearning graph.

**Figure 4:** Machine learning training process.

**Figure 5:** Metalearning training process.

**Table 1:** The research direction of metalearning in big data.

Research directions	Application scenarios	Research content	Learning objects	Advantages	Disadvantages
Classifier	Data prediction	Decision tree Logistic regression Naive Bayes Neural networks	Classification model with metafeatures	High prediction accuracy	Poor performance in schemes with strong indicator dependence

Metric	Few-shot learning	Relation network [30] Neural network [30] Prototypical network [31] Siamese neural network [32]	Metric space	Learning in space is efficient	Not applicable to regression and reinforcement learning

Optimizer	Finding the best strategy	Matching network [33] Graph neural network [34] Gradient descent [36] Curvature information matrix [37]	Optimizer	Metalearner can independently design an optimizer to complete new tasks	High optimization cost

**Table 2:** Specific analysis of the application of metalearning in the field of artificial intelligence.

Fields	Reasons for the rise	Specific application scenarios	Advantages
Few-shot learning	Limitations of dataset size	Face recognition [40] Classification [41, 42] Target detection [43, 44] Video synthesis [40]	Low dependence on sample size Strong generalization

Robot learning	The backwardness of robot operation skills	Imitation learning [49] Cross-domain learning [50] Quickly adapting online [51]	Improve the efficiency of autonomous learning by robots

Unsupervised learning	Poor performance of unsupervised learning algorithms	Distribution of unsupervised problems [52] Noise training [53]	Simplifying unsupervised learning to supervised learning Ability to learn from labeled data

Intelligent medicine	Slow progress in the medical field	Medical image processing [54] Drug discovery [56] Cancer detection [57] Medical vision question answering [58] Skin lesion segmentation tasks [60]	Predicting the specific behavior of molecules Ability to learn to weigh support samples

**Table 3:** Challenges and countermeasures of metalearning.

	Technical aspects	Application aspects
Specific problem	Costly Poor learning ability for complex tasks Single learning method of metaknowledge	Difficulty in obtaining data Inconsistent task distribution
Response plan	Improving model training performance Studying the continuity of action execution Metaknowledge combination learning	Building a training task database Learning from the experience of other algorithms [67–69]

## Data Availability

The data used to support the findings of this study are available from the corresponding author upon request.
